The article "Effects of LncRNA-HOST2 on cell proliferation, migration, invasion and apoptosis of human hepatocellular carcinoma cell line SMMC-7721" was retracted in 2021. Reasons: signs of a paper mill; concerns about the images.

# Effects of LncRNA-HOST2 on cell proliferation, migration, invasion and apoptosis of human hepatocellular carcinoma cell line SMMC-7721

**DOI:** 10.1042/BSR20160532

**Published:** 2017-04-20

**Authors:** Run-Tian Liu, Jing-Lin Cao, Chang-Qing Yan, Yang Wang, Cong-Jing An, Hai-Tao Lv

**Affiliations:** 1 Department of Hepatobiliary Surgery, The Second Hospital of Hebei Medical University, Shijiazhuang 050051, P.R. China; 2 Department of Hepatobiliary Surgery, The Third Hospital of Hebei Medical University, Shijiazhuang 050051, P.R. China; 3 Medical Examination Center, The Second Hospital of Hebei Medical University, Shijiazhuang 050051, P.R. China

**Keywords:** Human ovarian cancer specific transcript 2, Hepatocellular carcinoma, Long noncoding RNA, Migration, Proliferation, SMMC-7721 cell line

## Abstract

The present study explored the effect of long non-coding RNA-human ovarian cancer-specific transcript 2 (LncRNA-HOST2) on cell proliferation, migration, invasion and apoptosis of human hepatocellular carcinoma (HCC) cell line SMMC-7721. HCC tissues and adjacent normal tissues from 162 HCC patients were collected. The HCC cell lines were assigned into the control group (regular culture), negative control (NC) group (transfected with siRNA) and experimental group (transfected with Lnc-HOST2 siRNA). Quantitative real-time PCR (qRT-PCR) was used to detect the expression of LncRNA-HOST2. Cell proliferation was detected by CCK-8 and colony-forming assays, cell apoptosis by flow cytometry and cell migration by Scratch test. Transwell assay was used to evaluate cell migration and invasion abilities. LncRNA-HOST2 expression in the HCC tissues increased 2–10 times than that in the adjacent normal tissues. Compared with the HL-7702 cell line, LncRNA-HOST2 expression in HepG2, SMMC-7721 and Huh7 cell lines was all up-regulated, but the SMMC-7721 cell had the highest Lnc-HOST2 expression. The LncRNA-HOST2 expression in the experimental group was down-regulated as compared with the control and NC groups. In comparison with the control and NC groups, cloned cells reduced, cell apoptosis increased, clone-forming ability weakened and inhibitory rate of colony formation increased in the experimental group. The cells migrating and penetrating into the transwell chamber were fewer in the experimental group than those in the control and NC groups. The experimental group exhibited slow wound healing and decreased cell migration area after 48 h. These findings indicate that LncRNA-HOST2 can promote cell proliferation, migration and invasion and inhibit cell apoptosis in human HCC cell line SMMC-7721.

## Introduction

Hepatocellular carcinoma (HCC) is a leading cause of cancer-related mortality worldwide with its incidence rapidly increasing in the recent years [1]. It is estimated that 1 million people are expected to die from HCC annually since this disease is easy to be confused with cirrhosis, posing a great challenge for the early diagnosis and resulting in a sharp increase in HCC patients [2,3]. Many factors may result in HCC, among which infection of hepatitis A virus (HAV) or hepatitis B virus (HBV) tops [4]. Moreover, chemical and biological factors including heredity, signalling pathway disorder and protein dysfunction can also lead to cell damage, which remains one of the important causes of HCC [5]. Therefore, it is very important to understand tumour characteristics, liver function and physiological condition from various aspects for the diagnosis and treatment of HCC.

The article "Effects of LncRNA-HOST2 on cell proliferation, migration, invasion and apoptosis of human hepatocellular carcinoma cell line SMMC-7721" was retracted in 2021. Reasons: signs of a paper mill; concerns about the images.

Long non-coding RNA (LncRNA) is defined as an endogenous RNA with molecules longer than 200 nt in length [6–8]. LncRNA is usually transcribed by RNA polymerase II and formed by fragmentation and modification of the precursor RNA [9]. It can target the local gene and the distal gene and mainly regulates gene expression at transcription and post-transcription levels [10]. Recently, a large number of LncRNAs have been discussed in mammalian genomes and LncRNA level was presumably functional in some biological events such as specific stages of cancer, indicating different expressions of specific LncRNAs could work as indicators of early cancer diagnosis [11,12]. Furthermore, many molecular studies found that numerous LncRNAs play key roles in the progression of colorectal cancer, prostate cancer, liver cancer and many other human solid tumours [13]. Human ovarian cancer-specific transcript 2 (HOST2) is a member of LncRNAs, 2.9 kb in length, without a significant open reading frame (ORF), and it was reported to be highly expressed in human ovarian cancer [13–15]. Transcriptomics analysis showed that LncRNA level in HCC tissues also showed abnormal expression patterns, samples including highly up-regulated in liver cancer (HULC) gene highly up-regulated in HCC tissues and LncRNA HEIH promotes tumour progression in HBV-related HCC and its expression level is associated with recurrence and survival of patients [16], suggesting that different LncRNA expression might be related with HCC [17,18]. However, there has been no relevant report on LncRNA-HOST2 expression in HCC. In the present study, LncRNA-HOST2 expressions in tumour and adjacent normal tissues of 162 HCC patients were detected for *in vivo* experiment. Moreover, HCC cell lines were used to measure the *in vitro* effect of LncRNA-HOST2 on cell proliferation, migration, invasion and apoptosis.

The article "Effects of LncRNA-HOST2 on cell proliferation, migration, invasion and apoptosis of human hepatocellular carcinoma cell line SMMC-7721" was retracted in 2021. Reasons: signs of a paper mill; concerns about the images.

## Materials and methods

### Ethics statement

All clinical data were obtained after the approval of the Clinical Management Committee of The Third Hospital of Hebei Medical University and all the patients signed informed consents before operation.

### Specimen collection

HCC tissues and adjacent normal tissues 5 cm away from the cancer lesion of 162 HCC patients were collected from patients who were admitted in The Third Hospital of Hebei Medical University from 2012 to 2014 with well-preserved clinical and pathological data. Patients received no preoperative adjuvant therapies such as radiotherapy, chemotherapy and radiofrequency ablation. Post-operative HCC specimens were confirmed by two experienced pathologists. The degree of tumour differentiation was determined by Edmondson–Steiner grading standards. Tumour staging was determined by the seventh edition of staging system of American Joint Committee on Cancer (AJCC) issued in 2010. After being taken out, tissue specimens were placed in liquid nitrogen and transferred to be preserved at –80°C within 15 min.

### Cell culture

HCC cell lines HepG2, SMMC-7721 and Huh7 as well as normal liver cell line HL-7702 were obtained from the Hepatobiliary Surgery Department, Laboratory of Xijing Hospital of the Fourth Military Medical University. Cells were inoculated in the 60-mm culture dish with RPMI 1640 medium containing 10% FBS (Gibco Company, Grand Island, NY, U.S.A.) and cultured in an incubator at 37°C with 5% CO_2_ and saturated humidity. After cells grew along the dish wall, the medium was changed every 1–2 days and 0.25% trypsin (Sigma–Aldrich Chemical Company, St. Louis, MO, U.S.A.) was used for digestion and subculture.

### Cell grouping

The LncRNA-HOST2 expression was detected in human HCC cell lines HepG2, SMMC-7721 and Huh7 as well as human normal liver cell line HL-7702, the cell line that exhibited the most significant difference in LncRNA-HOST2 expression compared with Huh7 was selected for further use. The cell was assigned into control group (regular culture), negative control (NC) group (transfected with siRNA) and experimental group (transfected with Lnc-HOST2 siRNA).

### Cell transfection

The sequences of targeted gene *LncRNA-HOST2* were determined using BLAST in GenBank. From the initiation codon in AUG, continuous sequence of AA was found and siRNA sequence was designed targeting at 19 base sequences on the 3′-end. With avoiding the initiation codon, 5′-end, 3′-end, UTR and nonsense sequence, the GC content of siRNA sequences should be 30–50%. The specific primer on CDS region was designed using Primer Express 2.0 software. The sense sequence of LncRNA-HOST2 siRNA was 5′-GACUAAACAAGGUCUUAAUTT-3′ and the antisense sequence was 5′-AUUAAGACCUUGUUUAGUCTT-3′. The NC sequence had the same composition with the target siRNA sequence but without obvious homology. The sense sequence of NC siRNA was 5′-UUCUCCGAACGUGUCACGUTT-3′ and the antisense sequence was 5′-ACGUGACACGUUCGGAGAATT-3′. The above-mentioned sequences were synthesized by Shanghai Sangon Biotech Co. Ltd. According to the LncRNA-HOST2 sequence, targets for RNA interference and NC were designed. The corresponding fragment was synthesized and inserted into lentiviral vector through the restriction sites of EcoRI and BamHI after annealing. Verified if the vector was successfully constructed and sequenced, results showed that targeted fragments were inserted into the expression vector. Quantitative real-time PCR (qRT-PCR) was used to detect the LncRNA-HOST2 expression for evaluating effects of siRNA silencing LncRNA-HOST2. Lipofectamine 2000 (Invitrogen Inc., Carlsbad, CA, U.S.A.) was used for transfection according to instructions. HCC cell line SMMC7-721 was inoculated in a six-well plate with a concentration of 3 × 10^5^ cells/ml. After transfection, cells were divided into control, NC and experimental groups. After transfection for 48 h, cells were under detection for LncRNA-HOST2 siRNA level.

The article "Effects of LncRNA-HOST2 on cell proliferation, migration, invasion and apoptosis of human hepatocellular carcinoma cell line SMMC-7721" was retracted in 2021. Reasons: signs of a paper mill; concerns about the images.

### qRT-PCR

TRIzol reagent (Invitrogen Inc., Carlsbad, CA, U.S.A.) was used for the extraction of RNA in tissues or cells in accordance with instructions. Then the ultraviolet spectrophotometer was used to detect OD_260/280_ value of RNA specimen to calculate RNA concentration, after which the specimen was preserved at –80°C for later use. According to nucleotide sequences of glyceraldehyde 3-phosphate dehydrogenase (GAPDH) and LncRNA-HOST2 in Genebank, primers were designed by BLAST and the sequences are shown in Table 1. Primers were synthesized by Invitrogen Company. The experiment was performed in accordance with procedures provided by reverse transcription kit of TransGen Biotech (Beijing, China). qRT-PCR was conducted with a total volume of 20 μl: 10 μl of 2× SYBR Green QPCR master mix, 0.3 μl of diluted Reference Dye, 0.2 μl of upstream primer (10 μmol/l), 0.2 μl of downstream primer (10 μmol/l), 0.3 μl of cDNA and 9 μl of diethyl pyrocarbonate (DEPC) water. The reaction conditions were: pre-denaturation at 95°C for 10 min for 1 cycle, denaturation at 95°C for 30 s, annealing at 58°C for 1 min, extension at 72°C for 30 s for a total of 40 cycles. GAPDH was used as the internal control. Solubility curve was used to evaluate the reliability of PCR results. The average *C*_T_ value (amplified power curve inflection point) was taken. Semi-quantificative analysis and calculation of relative expression of the target gene were performed with 2^−^^ΔΔ*C*^_T_.

The article "Effects of LncRNA-HOST2 on cell proliferation, migration, invasion and apoptosis of human hepatocellular carcinoma cell line SMMC-7721" was retracted in 2021. Reasons: signs of a paper mill; concerns about the images.

**Table 1:** Primer sequences

PCR primers sequence	Forward (5′–3′)	Reverse (5′–3′)
LncRNA-HOST2	GGACAGGTCCCTTGTTTCAA	CTGGTCTTTCCTTGCCTCTG
GAPDH	CCACCCATGGCAAATTCCATGGCA	TCTAGACGGCAGGTCAGGTCCACC

### CCK-8 assay

SMMC-7721 cells in logarithmic growth phase were inoculated into a 96-well plate with every well containing 20000 cells. Cells were kept in the incubator with 5% CO_2_ overnight at 37°C. Before adding CCK-8, the medium was changed. For every well, 90 μl of medium and 10 μl of CCK-8 were added. The dish was kept in the incubator with 5% CO_2_ at 37°C for 1–2 h. The microplate reader was used for determination of OD value at 450 nm. The cell proliferation inhibition rate = (OD value of the experiment group – OD value of the control group)/OD value of the control group × 100%. The OD values were detected after culturing for 0, 24 and 48 h.

### Flow cytometry

The BD Annexin V-EGFP kit (Becton, Dickinson and Company, NJ, U.S.A.) was used for the experiment. SMMC-7721 cells were seeded in a six-well plate at a density of 2 × 10^5^ cells/well and processed after 24 h. The supernatant was collected in a 5-ml collection tube and cells were digested with 400 μl of trypsin. When cells turned to be round,the samples were centrifuged at 2000 rpm for 5 min, and the precipitate was collected followed by washing with 5% BSA(dissolved in PBS) twice. Then samples were centrifuged at 2000 rpm for 5 min, and the precipitate was collected followed by washing with 5% BSA (dissolved in PBS) twice. The supernatant was discarded, and the cells were resuspended in 300 μl of 5% BSA (PBS) and added with 700 μl of absolute ethanol for fixing. Cells were placed at –20°C for 24 h and centrifuged at 2000 rpm for 5 min. After that, FITC-Annexin V staining was conducted: cells were washed with 1 ml of PBS once, resuspended with 100 μl PBS and added with 1 μl of 10 mg/μl RNase A for incubation at 37°C. Then, 300 μl of 50 μg/μl PI was added for 20 min for detection. For PI staining, samples were washed with 2% BSA (PBS) twice and after removing supernatant, 500 μl of binding buffer was added for collecting cell suspension. Then, 5 μl of Annexin V-EGFP and 5 μl of PI were added, and the samples were preserved in the dark at room temperature for 5–15 min. BD FACS Flow Cytometry (Becton, Dickinson and Company, NJ, U.S.A.) was used for analysis.

### Clone-forming assay

Logarithmic growth phase SMMC-7721 cells were collected. Cells were fully dispersed for cell suspension. For the six-well plate, 100–200 cells were inoculated in each well. When visible clone appeared in the dish, the culture was terminated. The cells were then washed with PBS and dried in the air. The cells were fixed with methanol and stained with Crystal Violet. The plate was inverted, on which a piece of transparent film with grids was overlaid for clone counting. The clone formation rate = (the clone number/the number of inoculated cells) × 100% and the clone formation inhibition rate = (1 – (clone formation rate of the experiment group/clone formation rate of the control group)) × 100%.

The article "Effects of LncRNA-HOST2 on cell proliferation, migration, invasion and apoptosis of human hepatocellular carcinoma cell line SMMC-7721" was retracted in 2021. Reasons: signs of a paper mill; concerns about the images.

### Scratch test

Logarithmic growth phase SMMC-7721 cells were collected. Five lines were evenly drawn with a mark pen by a ruler on the outside bottom of the six-well plate with an interval of 0.5–1 cm. A total of 2 × 10^6^ SMMC-7721 cells were inoculated in the six-well plate and cultured to 90% fusion state. The cells were cultured in serum-free medium for starvation for 24 h. A 10-μl pipette tip was used to scratch the plate with a pattern of two lines perpendicular to each other. After 48 h of culture, the scratch healing was observed under the microscope and photographed. After cells were cultured for 0 h and 48 h, the area of the blank space was calculated. Then the migration area was calculated, after which changes of migration areas in all groups were compared. Migration area = blank space area (0 h) – blank space area (48 h).

### Transwell assays

SMMC-7721 cells in logarithmic growth phase were collected for cell suspension. Cell density was adjusted to 1 × 10^5^ cells/ml and 100 μl of cell suspension was added into the Transwell chamber. Then, 800 μl of medium (with transfection complexes or NC) was added into the 24-well plate in the lower chamber. Transwell chamber was removed after culture for 24 h. After being washed with PBS, cells were fixed with formalin. Then, a cotton swab was used to wipe upper cells of the microporous membrane and cells were stained with Crystal Violet. Under an inverted microscope, the image was magnified 200 times to count the number of cells in each field, in which cells were moved to the lower layer of the microporous membrane. In every specimen, five visual fields were counted and the whole assay was repeated three times. In the invasion experiment, 50 mg/l Matrigel (Sigma–Aldrich Chemical Company, St. Louis, MO, U.S.A.) diluent (1:8) was used to coat the upper chamber wall of the bottom membrane of the Transwell chamber (Corning Co., Ltd., Beijing, China), which was then dried in the air at 37°C. The residual liquid in the plate was cleaned out. Then, 50 μl of serum-free culture medium containing 10 g/l BSA was added in each well. Cells were cultured at 37°C for 30 min. The subsequent procedures were the same with those in the migration assay.

The article "Effects of LncRNA-HOST2 on cell proliferation, migration, invasion and apoptosis of human hepatocellular carcinoma cell line SMMC-7721" was retracted in 2021. Reasons: signs of a paper mill; concerns about the images.

### Statistical analysis

The data were analysed by SPSS 21.0 statistical software. The measurement data were expressed as mean ± S.D. For comparisons of normal distribution, *t* test was used. One-way ANOVA was used for comparisons among groups. The count data were expressed in percentage or rate and tested by chi-square test. *P*<0.05 was considered statistically significant.

## Results

### Relative expressions of LncRNA-HOST2 in HCC tissues and adjacent normal tissues and among HepG2, SMMC-7721, Huh7 and HL-7702 cell lines

The qRT-PCR was used to detect *LncRNA-HOST2* mRNA expressions in HCC tissues and adjacent normal tissues. Results showed that the expression of LncRNA-HOST2 in HCC tissues was up-regulated by approximately 2–10 times. When the LncRNA-HOST2 expression in HCC tissues was lower than two times of adjacent normal tissues, it was considered as low expression, and the LncRNA-HOST2 expression higher than two times was considered high expression. In 162 cases of HCC tissues, there were 87 cases of high expression (53.70%) and 75 cases of low expression (46.30%). Both high expression and low expression of LncRNA-HOST2 in HCC tissues were higher than those in adjacent normal tissues (all *P*<0.05) (Figure 1A). Analysis of the relation between LncRNA-HOST2 high or low expression and HCC clinicopathological features showed that LncRNA-HOST2 expression was not related to gender, age or level of animal protein factor (APF) (all *P*>0.05), while correlated with the size, quantity, distant metastasis and AJCC staging and differentiation degree of the tumour (all *P*<0.05) (Table 2 and Figure 2). qRT-PCR results showed that compared with the HL-7702 cell line, LncRNA-HOST2 expression in HepG2, SMMC-7721 and Huh7 cell lines was all up-regulated (all *P<*0.05), but the SMMC-7721 cell had the highest LncRNA-HOST2 expression, therefore, the SMMC-7721 cell was used for further analysis. (Figure 1B).

**Figure 1:** Expressions of LncRNA-HOST2 in the tissues and HCC cell lines detected by qRT-PCR (**A**) Relative expression of LncRNA-HOST2 in HCC tissues and adjacent normal tissues (when the LncRNA-HOST2 expression in HCC tissues was lower than two times of adjacent normal tissues, it was considered as low expression, and when the LncRNA-HOST2 expression was higher than two times, it was considered high expression); (**B**) Relative expression of LncRNA-HOST2 in HepG2, SMMC-7721, Huh7 and HL-7702 cell lines; ^*^P<0.05 compared with the HL-7702 cell line.

**Table 2:** Relationship between the LncRNA-HOST2 expression and clinicopathological features of HCC patients (*n*=162)

Feature	*n*	LncRNA-HOST2		*P*	OR (95% CI)
		High expression (*n*=87)	Low expression (*n=*75)		
Gender				0.549	1.323 (0.528–3.316)
Male	141	77	64		
Female	21	10	11		
Age (years)				0.176	1.535 (0.824–2.860)
<50	87	51	36		
≥50	75	36	39		
Tumour size				0.001	2.991 (1.572–5.690)
<5 cm	72	28	44		
≥5 cm	90	59	31		
Tumour number				<0.001	1.535 (0.824–2.860)
Single	89	30	59		
Multiple	73	57	16		
APF level (ng/ml)				0.374	1.324 (0.712–2.462)
<400	86	49	37		
≥400	76	38	38		
Distant metastasis				0.031	1.984 (1.059–3.715)
No	76	34	42		
Yes	86	53	33		
TNM staging				0.002	2.726 (1.442–5.156)
III + IV	84	55	29		
I + II	78	32	46		
Differentiation degree				0.012	2.229 (1.187–4.186)
Low	82	52	30		
High/middle	80	35	45		

CI, confidence interval; OR, odd ratio; TNM, tumour node metastasis.

The article "Effects of LncRNA-HOST2 on cell proliferation, migration, invasion and apoptosis of human hepatocellular carcinoma cell line SMMC-7721" was retracted in 2021. Reasons: signs of a paper mill; concerns about the images.

**Figure 2:** Correlations of relative expressions of LncRNA-HOST2 with the clinicopathological characteristics of HCC patients (**A**) Relative expressions of LncRNA-HOST2 in HCC patients with different tumour sizes detected by qRT-PCR; (**B**) Relative expressions of LncRNA-HOST2 in HCC patients with different tumour numbers detected by qRT-PCR; (**C**) Relative expressions of LncRNA-HOST2 in HCC patients with differing degrees of metastasis detected by qRT-PCR; (**D**) Relative expressions of LncRNA-HOST2 in HCC patients with different stages detected by qRT-PCR; (**E**) Relative expressions of LncRNA-HOST2 in HCC patients with differing degrees of differentiation detected by qRT-PCR.

### Effect of siRNA transfection on LncRNA-HOST2 expression of the SMMC-7721 cell line

siRNA was synthesized and used for cell transfection. LncRNA-HOST2 was targeted and its expression was inhibited. The qRT-PCR result showed that compared with control group and NC group, LncRNA-HOST2 expression in the experimental group was down-regulated (both *P*<0.001). There was no significant difference in LncRNA-HOST2 expression between the NC and control groups (*P*>0.05) (Figure 3).

**Figure 3:** Relative expressions of LncRNA-HOST2 in SMMC-7721 cells among the control, NC and experimental groups detected by qRT-PCR (**A**) Electrophoresis of LncRNA-HOST2 mRNA in SMMC-7721 cells among the three groups; (**B**) Grey value analysis for (A); (1): control group; (2): NC group; (3): experimental group; ***P<0.001 compared with the control or NC groups.

### Effect of LncRNA-HOST2 expression on cell proliferation of the SMMC-7721 cell line

OD values of 0, 24 and 48 h were used for drawing the growth curve. CCK-8 assay found that there was no significant difference of T_0_ absorbance between the experimental group with the negative and NC groups (*P*>0.05), while after inhibiting HOST2 expression for 24 h and 48 h, proliferation ability of cells was suppressed in comparison with the control group and the NC group (*P*<0.05) (Figure 4). The *in vitro* cloning assay results showed that the number of cloned cells declined (Figure 5C), colony formation ability weakened (Figure 5A) and inhibition rate of colony formation increased in the experimental group (*P*<0.001) (Figure 5 B). There was no significant difference of clone ability between the NC and control groups (*P*>0.05).

The article "Effects of LncRNA-HOST2 on cell proliferation, migration, invasion and apoptosis of human hepatocellular carcinoma cell line SMMC-7721" was retracted in 2021. Reasons: signs of a paper mill; concerns about the images.

**Figure 4:** Effect of LncRNA-HOST2 expression on the proliferation of SMMC-7721 cells at 0, 24 and 48 h detected by CCK-8 assay *P<0.05 compared with the control group or the NC group.

**Figure 5:** Effect of LncRNA-HOST2 expression on the proliferation of SMMC-7721 cells evaluated by clone-forming assay (**A**) Clone formation rate; (**B**) Clone inhibition rate; (**C**) Clone number; ***P<0.001 compared with the control group or the NC group; *n*, replicate numbers.

### Effect of LncRNA-HOST2 expression on cell cycle of the SMMC-7721 cell line

There was no significant difference of cell cycle between the NC and control groups (*P*>0.05). In comparison with the control and the NC group, cells in G_0_/G_1_-phases were increased (*P*<0.05), while no significant difference of cells in G_2_/M-phases was observed in the experimental group (both *P*>0.05). However, cells in S-phase of the experimental group were markedly decreased (*P*<0.05). Results showed that with suppressed LncRNA-HOST2 expression, SMMC-7721 cells were blocked from G_0_/G_1_-phases to S-phase, which indicated that cell proliferation ability was inhibited (Figure 6).

**Figure 6:** Effect of LncRNA-HOST2 expression on cell cycle of SMMC-7721 cells detected by flow cytometry (**A**) Effect of LncRNA-HOST2 expression on cell cycle of SMMC-7721 cells (**B**) Cell-cycle distribution of SMMC-7721 cells in three groups; *P<0.05 compared with the control group or the NC group.

### Effect of LncRNA-HOST2 expression on cell migration and invasion of the SMMC-7721 cell line

Transwell assay showed that compared with the NC and control groups, the migration and invasion abilities in the experimental group were decreased (*P*<0.001). There was no significant difference between the NC and control groups (*P*>0.05) (Figure 7). The results demonstrated that inhibiting LncRNA-HOST2 expression suppressed migration and invasion of HCC cell line SMMC-7721. Scratch test (Figure 8) suggested that after culture for 48 h, scratches of the experimental group healed slowly and the area of cell migration reduced (*P*<0.01). While scratches of the control group and the NC group were basically covered by cells and there was no significant difference of migration areas between the two groups (*P*>0.05), indicating that inhibition of LncRNA-HOST2 expression could reduce migration and invasion abilities of SMMC-7721 cells.

The article "Effects of LncRNA-HOST2 on cell proliferation, migration, invasion and apoptosis of human hepatocellular carcinoma cell line SMMC-7721" was retracted in 2021. Reasons: signs of a paper mill; concerns about the images.

**Figure 7:** Effect of LncRNA-HOST2 expression on cell migration and invasion of SMMC-7721 cells detected by Transwell assays (**A**) Migration and invasion patterns using Transwell chamber; (**B**) Numbers of cell migration; (**C**) Numbers of cell invasion; ***P<0.001 compared with the control group and the NC group; *n*, visual fields’ number counted in each group.

**Figure 8:** Effects of LncRNA-HOST2 expression on cell migration of SMMC-7721 cells detected by Scratch test (**A**) Cell migration observed under the microscope before and after suppressed LncRNA-HOST2 expression; (**B**) Comparison of cell migration areas among control group, NC group and experimental group before and after suppressed LncRNA-HOST2 expression; ***P<0.001 compared with the control group or the NC group; *n*, number of visual fields photographed by microscope in each group.

## Discussion

In the present study, *in vivo* and *in vitro* experiments both verified the effects of LncRNA-HOST2 expression on development and progression of HCC. Initially, the results of experiments on clinical specimens showed that the expression of HOST2 increased in HCC tissues and was related to the size, number, metastatic ability and differentiation degree of the tumour. Also, results of experiments on cells verified that the increased expression of HOST2 increased cell proliferation, as well as cell migration and invasion, which was consistent with previous study that the increased expression of LncRNA in HCC tissues was mainly related to the invasion of HBV [19]. Multiple LncRNAs are demonstrated to be correlated to HCC, Wang et al. [20] indicated that LncRNA-UCA1 up-regulation promotes HCC progression accompanied by *miR-216b* inhibition, and Lv et al. showed that LncRNA H19 and *miR-675* inhibition contributes to migration and invasion of HCC [21]. *HOST2* is a novel gene that contains plentiful copies of retroviral-related sequences [14]. However, limited evidence have shown the relationship between HOST2 expression and HCC. According to related researches, HOST2 expression was closely related to increased level of claudin in the process of cancer development [22,23]. HOST2, as a member of the HOST family, is associated with the proliferation and differentiation of tumour cells. It has been confirmed that HOST family is associated with gene function of proteoglycan link protein (LP) and *LP* gene can regulate the formation of extracellular matrix (ECM) [24], which is beneficial for intercellular coupling for promoting cell differentiation. Meanwhile, the HOST family also regulates the function of metastasis molecule coded by SLC34A2. It was reported that SLC34A2 had high expression in ovarian cancer cells, which promoted proliferation, mobility and differentiation of cells [25].

The article "Effects of LncRNA-HOST2 on cell proliferation, migration, invasion and apoptosis of human hepatocellular carcinoma cell line SMMC-7721" was retracted in 2021. Reasons: signs of a paper mill; concerns about the images.

In addition, HOST2 can regulate proliferation, metastasis and invasion of tumour cells with special regulation means. It is known that the major role of LncRNAs in disease progression are the mechanisms by which these RNAs seek their targets and control the epigenetic trajectory contributing to their ontogeny [26,27]. Moreover, the oncogenic activity of some LncRNAs could be attributed to miRNAs [28]. Gao et al. [15] have pointed out that LncRNA H19 can act as a molecular ‘sponge’ for *miR-let-7b*, and in the regulation process of HOST2, the level of *miR-let-7b* was regulated, which inhibited the activity of let-7b and increased mRNAs and protein levels of high-mobility group including AT-hook 2 (HMGA2), c-Myc, Dicer and Imp3, thus inducing cell metastasis and invasion in ovarian cancer [15]. Among these factors, HMGA2, c-Myc and Imp3 are related to metastasis and infection of tumour cells. HMGA2 is able to regulate multiple pro-metastatic factor genes and improve the process of tumour cell metastasis [29]. c-Myc can activate formation and metastasis of tumours [30], directly activate *Lin28* gene and then further inhibit the level of let-7b, resulting in deterioration in cancer progression [31]. Imp3 is often expressed in a variety of invasive cancer cells and can regulate invasion-related genes after they are transfected, thus enhancing the movement ability and infectivity of tumour cells [32]. As for Dicer, it is an important synthesis-related factor of miRNA and relates to tumour cell activities [33]. In addition, the retinoblastoma protein (pRb) and the transcription factor p53 are two major tumour-suppressor pathways functioning in control of cellular responses to potentially oncogenic stimulants, and distinct LncRNAs are involved in these pathways that control cell-cycle progression and survival [34,35]. The let-7 family members can target critical cell-cycle regulators such as CDK6 thus inducing cell cycle arrest at the G_1_-phase [36]. All in all, HOST2 can directly or indirectly regulate proliferation, growth and metastasis-related factors and ultimately promote the further deterioration of cancer. We speculate that the mechanism involved in HCC might be similar to this, but detailed monocular mechanism needs be verified by further researches.

Consequently, our study provides evidence that LncRNA-HOST2 can promote cell proliferation, migration and invasion and inhibit cell apoptosis in human HCC cell line SMMC-7721. Although detection of LncRNA HOST between HCC tissues and adjacent normal tissues was performed, no follow-up on prognosis of HCC patients was conducted, which requires validation and confirmation in future studies for the effects of HOST2 on pathological progression of HCC and patients’ survival.

The article "Effects of LncRNA-HOST2 on cell proliferation, migration, invasion and apoptosis of human hepatocellular carcinoma cell line SMMC-7721" was retracted in 2021. Reasons: signs of a paper mill; concerns about the images.

## Abbreviations

AJCC: American Joint Committee on Cancer
APF: animal protein factor
GAPDH: glyceraldehyde 3-phosphate dehydrogenase
HBV: hepatitis B virus
HCC: hepatocellular carcinoma
HMGA2: high-mobility group including AT-hook 2
HOST2: human ovarian cancer specific transcript 2
LncRNA: long non-coding RNA
LP: link protein
NC: negative control
qRT-PCR: quantitative real-time PCR
